RETRACTED

# The deformation monitoring of foundation pit by back propagation neural network and genetic algorithm and its application in geotechnical engineering

**DOI:** 10.1371/journal.pone.0233398

**Published:** 2020-07-01

**Authors:** Jie Luo, Ran Ren, Kangde Guo

**Affiliations:** 1 Department of Architecture and Civil Engineering, City University of Hong Kong, Kowloon, HongKong, China; 2 Water environment branch, China Metallurgical Group Corporation Huatian Company. Nanjing, China; 3 Department of Business administration, Macau University of Science and Technology, Taipa, Macau, China; University College London, UNITED KINGDOM

## Abstract

The objective is to improve the prediction accuracy of foundation pit deformation in geotechnical engineering, thereby provide early warning for engineering practice. The digital close-range photogrammetry is used to obtain monitoring data. The error compensation method is used to optimize the center of the monitoring point. Aiming at the limitations of back propagation neural network (BPNN), a genetic algorithm (GA)-optimized BPNN algorithm is proposed. Then, the optimized algorithm is applied to predict the deformation and displacement of foundation pits from three aspects, i.e., simple horizontal displacement, simple longitudinal displacement, and the combination of horizontal and longitudinal displacements. Meanwhile, the time domain, space domain, and time-space domain are used as input features to compare the prediction results of the BPNN model and the GA-optimized BPNN model. Finally, the GA-improved BPNN is compared with the Support Vector Regression (SVR) model and Random Forest (RF) model. The results show that the prediction result, obtained by simultaneously using horizontal displacement and longitudinal displacement as input features, has smaller errors; also, the actual output is closer to the expected output. Compared with the prediction result with time domain and space domain as input features, the prediction result with time-space domain as input features is closer to the expected output. Taking the combination of time and space domains as input features, compared with the BPNN model, the GA-optimized BPNN model has a lower Root Mean Squared Error (RMSE) value (0.0163), a larger Index of Agreement (IA) value (0.9800), and a shorter training time (7.08 s). Compared with the SVR model and RF model, the GA-improved BPNN model has a lower Root Mean Squared Error (RMSE) value (0.0211), a larger Index of Agreement (IA) value (0.9706), and shorter training time (7.61 s). Therefore, the foundation pit deformation prediction model based on BPNN and GA has strong prediction ability, which can be popularized and applied in similar geotechnical engineering.

RETRACTED

## 1. Introduction

Recently, as urbanization progresses in China, the exploitation and utilization of underground space continue to develop. Therefore, geotechnical engineering has become a major topic in urbanization construction. The number of geotechnical engineering projects has been increasing. Geotechnical engineering is developing in the direction of larger and deeper, whose theory and technology are also advancing with the times [1]. In geotechnical engineering, the safety of foundation pits is an essential guarantee for the implementation of subsequent projects. Once an accident occurs, the economic losses, casualties, and social impacts are immeasurable [2]. Therefore, the safety construction problem in foundation pit engineering has become a critical problem in contemporary urban construction. Traditional deformation monitoring methods have vital effects in the early warning of foundation pit problems. However, limitations, such as accurate positioning, prediction, and early warning, still exist [3]. While constructing the foundation pits, only after comprehensive monitoring of the surrounding soil and supporting structure can a systematic understanding of the project be ensured; therefore, the geotechnical engineering will go smoothly [4]. As one of the important branches of modern technology, artificial intelligence (AI) algorithms have achieved fruitful results in engineering application. Therefore, applying AI algorithms to the deformation monitoring of modern foundation pit construction projects is critically significant. Neural network algorithm is one of the hot spots in AI algorithms. Among them, back propagation neural network (BPNN) can approximate any function theoretically, and the basic structure of the network is composed of non-linear change units, which has strong non-linear mapping ability; thus, it is widely used in biology, chemistry, agriculture, engineering, and other fields. At present, scholars have applied it to the deformation monitoring of foundation pits. Because BP neural networks have the disadvantage of being easily trapped in locally optimal solutions, in recent years, there has been an endless stream of corresponding improvements to BP neural networks. Based on the theory of BPNN, Cui and Jing (2019) built a model for predicting geotechnical parameters by using the geological engineering database as the development basis, as well as analyzing the material features, sediment distribution, and other parameters of geotechnical engineering [5]. Zhang et al. (2019) proposed a combination prediction model through discrete gray Verhulst model and BPNN. The model had high prediction accuracy and stability for predicting the settlement of foundation pits [6]. Currently, most foundation pit monitoring mainly considers the monitoring instrument layout, data acquisition, and report submission; however, it often does not consider monitoring data analysis and feedback, thereby cannot make corresponding early warnings in combination with the factors affecting the pit and the surrounding environment. As a result, it takes a lot of manpower and material resources but cannot obtain required analysis feedback, nor can it optimize the design of the subsequent construction of the foundation pit. In most of the foundation pit deformation monitoring methods based on neural networks, the input features only consider the time series, without combining other influencing factors. In addition, local optimization occurs in the BPNN. Therefore, it is necessary to optimize it, thereby improve the prediction effect.

RETRACTED

In summary, the monitoring position of the foundation pit supporting directly affects the accuracy and reliability of subsequent geotechnical engineering. Therefore, its accurate positioning is necessary. To accurately predict the deformation of the foundation pits and reduce the losses due to the safety issues, this study takes the foundation pit project in X city as an example. Through the BPNN and GA, the identification and accuracy of the pit supporting monitoring point positioning are improved. The innovation of this study is to comprehensively consider the characteristics and factors in foundation pit construction, and to improve the method of foundation pit deformation monitoring based on BPNN. This study has vital theoretical and practical values for the early warning of engineering practice.

## 2. Method

### 2.1 Identification and positioning of monitoring point center

Foundation pit monitoring is an essential link in safe geotechnical engineering. It is also the technical support and vital guarantee for the safe implementation of the project. During the construction of foundation pits, deformation is usually caused by various factors. This study takes a foundation pit project in X city as an example for deformation monitoring. First, the monitoring points and reference points are arranged. The surrounding environment, geological conditions, and geographical and climate factors are considered to arrange the top side slope monitoring point, the adjacent road monitoring point, and monitoring points of surrounding pipelines and groundwater table. After the arrangements are complete, the initial value is collected 3 times before the foundation pit excavation. Daily monitoring is started from the excavation day of the foundation pit. Meanwhile, according to the needs of monitoring the horizontal displacement and longitudinal displacement of the project, three reference points are set in a relatively flat area outside the foundation pit. The second monitoring is performed one month after the construction. The subsequent monitoring is performed once every one month thereafter. With the *Code for Design of Building Foundation* as the standard for controlling the deformation of structures, the relevant allowable values for the deformation of different structures during the construction are formulated [7]. The measuring instruments include DINI03 surveyor’s level (Trimble Navigation, USA) and GTS102N total station (Beijing Topcon, China). In addition, this study also uses digital close-range photogrammetry technology, and the camera used is EOS 5D Mark IV (Canon, Japan).

RETRACTED

Currently, the report data of foundation pit monitoring only have a simple feedback function. Further researches on the errors between the placement of measuring instruments, the coordinates of the target point measured by photography, and the coordinates of the actual target during the monitoring of the pit are rare. To improve the measurement accuracy, this study optimizes the monitoring point center by error compensation method [8]. An error compensation method of multi-dimensional feature camera calibration is used to determine the center positioning of the foundation pit monitoring point. Images of the foundation pit taken from the monitoring points are collected by the EOS 5D Mark IV camera. Key points are selected from each image, whose color features, local Gabor features, and global associated features are extracted. The actual error between each key point coordinate and its ideal position coordinate is calculated. The SVMLight tool is used to perform support vector regression (SVR) model training, and a model file for the calculation of key point compensation values is obtained [9]. In addition to reducing the camera calibration error, the center position needs to be optimized by multi-target center optimization technology based on rough K-means to improve the recognition accuracy [10]. The K-means algorithm is used to find the robustness of the clustering center, thereby optimizing the positioning of the monitoring center of the foundation pit and obtaining the optimal coordinates [11]. The measured target images are converted into image signals, which are uploaded to an image processing system and be converted into digital signals. Then, the digital signals are converted into grayscale images from the binary grayscale. The rough K-means clustering algorithm is as follows:

    *C*_*j*_ = *random*(U), // where: j = 1:1:n, C_j_ is the set of initial cluster center, U is the data set

    for i = l to m do // m is the number of elements in U

        for j = l to n do // n is the number of elements

            *d* = |*X*_*i*_−*C*_*j*_| // d is the distance from the current element *X*_*i*_ to a designated cluster center *C*_*j*_

        if *d*<*d*_min_ &&*d*<*c* then // *d*_*min*_ is the smallest distance, c is the threshold for setting the boundary area

            *d*_min_ = *d*

            *W*_*j*_ = *X*_*i*_∪*W*_*j*_ // *W*_*j*_ is the division of *j* sets

        end if

    end for

   end for

   for j = l to n do

      *R*_*j*_ = *getRadius*(*W*_*j*_)

      for i = l to m do

         $f_{j}^{i}=getlmpact\left(X_{i},r_{j}\right)$

         Update Center ($f_{i}^{j},W_{j}$)

      end for

   end for

      t = t+1 // t is the iteration counter since 0

   if t>T || is Stable (V) then

      end;

   else

      goto line2

   end if

First, the cluster center is initialized, and the function is *random ()*. Then, the selected samples are divided according to the cluster center, and the class center is updated. When the cluster becomes stable or reaches the preset number of iterations threshold, the iteration ends; otherwise, it continues to jump to line 2 of this algorithm.

RETRACTED

Monitoring point A is taken as an example, whose original foundation pit image and the optimized foundation pit image are compared to verify the feasibility of the combination of digital close-range photogrammetry and error compensation in optimizing the monitoring point center.

### 2.2 BPNN algorithm

The BPNN includes two stages of operation. First, the signals are propagated forward from the input layer to the output layer, during which the signals pass through the hidden layer. Second, the signals are propagated backward from the output layer to the input layer, during which the signals pass through the hidden layer. The weight and error of the hidden layer to the output layer are adjusted successively, as well as the weight and error of the input layer to the hidden layer. When the error after the network training is less than the set threshold, the neural network parameter training ends [12].

The signal input of the *i*-th node in the network structure is shown in Eq (1):

$${\mathrm{net}}_{i}=\sum_{j=1}^{M}w_{ij}x_{j}+\theta_{i}$$ (1)

Where: *w*_*ij*_ represents the weight of the *j*-th node in the input layer to the *i*-th node in the hidden layer, *x*_*j*_ represents the input signal of the *j*-th node in the input layer, and *θ*_*i*_ represents the threshold of the *i*-th node in the hidden layer.

The output of the *i*-th node in the hidden layer is shown in Eq (2):

$$o_{i}=\phi \left({\mathrm{net}}_{i}\right)$$ (2)

Where: *ϕ*( ) is the excitation function of the hidden layer.

RETRACTED

After the hidden layer is passed to the output layer, the input of the *k*-th node in the output layer is as shown in Eq (3).

$${\mathrm{net}}_{k}=\sum_{i=1}^{q}w_{ki}\phi \left({\mathrm{net}}_{i}\right)+a_{k}$$ (3)

Where: *w*_*ki*_ is the weight of the *i*-th node in the hidden layer to the *k*-th node in the output layer, and *a*_k_ is the threshold of the *k*-th node in the output layer.

The output of the *k*-th node in the output layer is shown in Eq (4).

$$o_{k}=\psi \left({\mathrm{net}}_{k}\right)$$ (4)

Where: *ψ*( ) is the excitation function of the output layer.

In back propagation, there are *p* training samples, and the sample error is as shown in Eq (5).

$$E_{p}=\frac{1}{2}\sum_{p=1}^{p}\sum_{k=1}^{L}{\left(T^{p}{}_{k}-O^{p}{}_{k}\right)}^{2}=\sum_{p=1}^{p}E_{p}$$ (5)

Where: *T*^*p*^_*k*_ represents the expected value of the *k*-th node, *L* is the total number of nodes in the network.

According to the gradient descent iterative method, the connection parameters in the network structure are modified. Further calculation can obtain the input layer weight correction value, the threshold correction value, the output layer weight correction value, and the threshold correction value of the BPNN.

### 2.3 Genetic algorithm and improved BPNN

BPNN also has some limitations, such as randomness in selecting original weights and thresholds, and being easy to fall into a local optimal solution. Meanwhile, genetic algorithm (GA) has better function optimization and search capabilities; however, compared with BPNN, its learning ability is poor [13, 14]. GA is a non-linear global optimization algorithm inspired by biological evolution mechanisms (survival of the fittest, crossover, and mutation). Starting from an initial population, it effectively achieves a stable and optimized breeding and selection process through individual genetics and mutation, retaining previously selected fitness function; otherwise, it will be eliminated. Compared with general optimization algorithms, GA does not depend on gradient information. It mainly works on encoded chromosomes and has the advantages of wide adaptive range, strong global search ability, high parallelism, and high scalability. The GA is not affected by other factors, and individuals are mainly evaluated based on the fitness function within the algorithm. Therefore, GA is easy to be combined with other algorithms to utilize the advantage of both. By combining GA and BPNN, GA simultaneously processes different individuals in the population and guide the search direction of the algorithm according to the principle of uncertainty. During the searching process, it effectively prevents convergence to the local optimal solution, thereby overcoming the shortcoming of BPNN, i.e., easily falling into a locally optimal solution. Therefore, this study combines BPNN and GA, which not only avoids the convergence to the local optimal solution but also improves the generalized fault tolerance of BPNN and the accuracy of convergence recognition.

RETRACTED

After the parameters of the BPNN and the GA are determined, the population and parameters are initialized. Meanwhile, the threshold and the weight of the neural network are combined and encoded. The GA is used to optimize the original weight of the BPNN, calculate the fitness function, and retain a higher degree of fitness. The crossover operation and mutation operation in the GA are performed on the individual chromosomes in the population, thereby generating the next generation of individuals. Until the number of generations reaches a fixed generation time or converges to a value, or the fitness value is less than the termination criterion, the generation is terminated. The optimal weight and threshold are obtained and used as the original weight and threshold of the BPNN. The BPNN is trained until the set value of error appear, and the final result is obtained.

### 2.4 Deformation monitoring method based on BPNN and GA

Deformation monitoring data of the horizontal displacement monitoring point B at the top of the side slope is selected. The previous 85% of the data samples are utilized as the training sample, and the last 15% of the data are used as the prediction sample. The monitoring sample data are normalized to [0.1, 0.9]. The normalized value of the sample is calculated by Eq (6).

$$X'=0.8\times \frac{X-X_{\min}}{X_{\max}-X_{\min}}+0.1$$ (6)

Where: *X*_max_ represents the maximum value in the sample data, and *X*_min_ represents the minimum value in the sample data.

Similarly, the final output value is de-normalized. The newff function in the neural network toolbox is used to build a new BPNN, as shown in Eq (7).

$$net=newff\left(PF,\left[S_{1}S_{2}\ldots S_{i}\right],\left\{{\mathrm{TF}}_{1}{\mathrm{TF}}_{2}\ldots {\mathrm{TF}}_{i}\right\},\mathrm{BTF},BLF,PF\right)$$ (7)

Where: PF represents the mean square error, *S*_*i*_ represents the number of units in the *i*-th layer, *Tf*_*i*_ represents the transfer function of the *i*-th layer, BTF represents a training function, and BLF represents a learning algorithm.

The original weight and threshold of the network are set. To prevent the neurons from entering the saturation state while the network is trained, the weight should not be too large. The train function is used to train the BPNN. When the training reaches a preset number of steps or the training error is smaller than a set threshold, the training is terminated, and the values are de-normalized. The normalized prediction samples are input and simulated by using a trained network, and the normalized results are obtained by de-normalizing.

RETRACTED

The prediction model is built by using the BPNN optimized by GA. First, the original weight and threshold of the BPNN are used as chromosomes and encoded. The optimal initial weights and thresholds are assigned to the BPNN through GA. The displacement deformation of the monitoring points of the foundation pit is predicted through the training of the BP network. The results are run in Matrix Laboratory (MATLAB) and the network normalized results are output.

The BPNN optimized by GA is used to predict the deformation and displacement of the foundation pit from the three aspects, i.e., simple horizontal displacement, simple longitudinal displacement, and horizontal-longitudinal displacement error, respectively.

### 2.5 Deformation prediction model of multi-order spatiotemporal foundation pit deformation

Both temporal and spatial features are vital features in the displacement prediction of monitoring points. Therefore, this study builds a multi-order spatiotemporal feature matrix to expand features from similar time domains to all time domains and from adjacent monitoring points to all monitoring points. The autocorrelation function is used to calculate the order correlation of the temporal features of the monitoring point B as in Eq (8). The order correlation of the spatial features is as shown in Eq (9).

$$p_{n}=\frac{1}{P-n}\sum_{i=1}^{P-n}\frac{h_{i}h_{i+n}}{H*H},\left(n=1,2,\ldots ,m\right)$$ (8)

Where: *P* represents the length of the time series data of the collected foundation pit, *h*_*i*_ represents the time-domain feature of the *i*-th monitoring, *H* represents the sum of all-time data, and *m* represents the order of the correlation coefficient.

$$q_{n}=\frac{1}{Q-n}\sum_{j=1}^{Q-n}\frac{s_{j}s_{j+n}}{S*S},\left(n=1,2,\ldots ,m\right)$$ (9)

Where: *Q* indicates the number of monitoring points of the foundation pit, *s*_*i*_ indicates the features of the *i*-th monitoring point, and *S* indicates the sum of the feature data of all monitoring points.

A time domain prediction model is built. The deformation monitoring data of monitoring point B is set. The past 5 days in the sample data are used as the time-domain feature input to predict the horizontal displacement in the future. The network training sequentially takes 5 samples of the time domain feature as sliding windows and maps them into a 1-day value. The previous 85% of the data is used as the training sample, and the last 15% of the data is used as the prediction sample.

RETRACTED

A space domain prediction model is built, the displacement of one day after the 10 monitoring points adjacent to monitoring point B is selected as a space domain feature input to predict the displacement of monitoring point B in the next day. The 85% of the previous data are used as training samples, and 15% of the data are used as prediction samples.

A prediction model combining both time domain and space domains is built. Deformation monitoring data of monitoring point B and its adjacent 10 monitoring points are selected. By taking the past 5 days of monitoring point B as the time domain feature input, and the displacement of the next 10 monitoring points one day later as the space domains feature input, the displacement of monitoring point B in the next day is predicted. Sequentially, 5 samples of the time domain feature are taken as sliding windows and maps them into a 1-day value. The previous 85% of the data is used as the training sample, and the last 15% of the data is used as the prediction sample.

The simulation values and the actual monitoring values of BPNN model and GA-optimized BPNN model are compared with the three cases of time domain, space domain and time-space domain. The Root Mean Squared Error (RMSE) and the Index of Agreement (IA) of the three prediction models, including the time domain prediction model, space domain prediction model, and time-space prediction model, are calculated, as shown in Eqs (10) and (11).

$$RMSE=\sqrt{\frac{\sum_{i=1}^{n}{\left(X_{o,i}-X_{p,}{}_{i}\right)}^{2}}{n}}$$ (10)

Where: *n* represents the total number of samples, *Xo*,*i* represents the actual value of the i-th sample, and *Xp*,*i* represents the predicted value of the *i*-th sample.

$$IA=1-\frac{\sum_{i=1}^{n}{\left(X_{o,i}-X_{p,}{}_{i}\right)}^{2}}{\sum_{i=1}^{n}{\left(\left|X_{p,}{}_{i}-\bar{X_{o}}\right|+|X_{o,i}-\bar{X_{o}}\right)}^{2}}$$ (11)

Where: $\bar{X_{o}}$ represents the average of all actual values in the sample.

The RMSE, IA, and training time are taken as the evaluation indicators of test results. In the actual measurement, the number of observations is always limited, and the true value is only replaced by the most reliable (optimal) value. RMSE is an indicator used to measure the deviation between the observed value and the true value. Therefore, RMSE indicates the quality of observations to a certain extent. The better the quality of observations is, the smaller the RMSE is. IA is used to judge the fitting effect of the model. The larger the value is, the better the fitting effect of the model is. Under the condition that the prediction accuracy is guaranteed, the shorter the training time of the model is, the faster the convergence speed of the model is.

RETRACTED

### 2.6 Comparison with other typical prediction methods

To further verify the reliability of this algorithm, it is compared with other classic prediction algorithms, including the SVR prediction algorithm [15] and the RF regression prediction method [16]. The horizontal displacement deformation of monitoring point B is predicted in MATLAB, and the results of the final regression prediction output are compared with the genetic algorithm-improved BP neural network model.

A Support Vector Machine (SVM) maps a set of linearly inseparable data into a higher-dimensional space through a non-linear transformation, thereby finding the optimal linear distinguishing plane for the samples in this space. This algorithm can minimize the risk and has obvious advantages in dealing with the number of small samples, obvious non-linear characteristics, and high-dimensional problems. The SVR prediction method is as follows. The combination of time domain and space domain features is used as the input of the SVR algorithm influencing factors. Deformation monitoring data of the horizontal displacement monitoring point B at the top of the side slope is selected. The previous 85% of the sample data is used as the training sample, and the last 15% of the data is used as the prediction sample. Relevant preprocessing is performed on the sample data. The kernel function of the algorithm is a Radial Basis Function (RBF). Through the particle swarm optimization algorithm, the kernel function parameters and penalty factors in the SVR algorithm are optimized to obtain the optimal kernel function parameters and penalty factors [17]. The k-cross validation algorithm is used to correlate the mean square error (MSE) [18]. If the requirements are met, follow-up operations are performed; otherwise, the optimal parameters are found again. An SVR prediction model of foundation pit deformation and displacement is established and predicted.

The RF model is composed of several independent decision trees, where each decision tree randomly selects samples and features to obtain multiple weak classifiers for local domain learning and combines them into a global strong classifier [19]. In the process of building the model, there are relatively few parameters that need to be adjusted, which only include the number of Classification And Regression Tree (CART) and split attributes. The RF regression prediction method is as follows. The deformation monitoring data of the monitoring point B of the foundation pit are obtained. The samples and features in the monitoring data sample of the foundation pit are randomly selected. The optimal segmentation feature and the optimal segmentation point are selected; thus, each group of training data is formed accordingly. The CART decision tree consists of a decision tree composed of RF prediction models and iteratively calculates the minimum loss function to vote. The final prediction result is the sum of the predictions of each decision tree and then averaged.

RETRACTED

## 3. Results and discussion

### 3.1 Identification and optimization results of monitoring point center

Taking the monitoring point A as an example, the original foundation pit image and the optimized foundation pit image are shown in Fig 1. The monitoring point center shown in the optimized foundation pit image is very close to the ideal monitoring point center. The changes in the horizontal and longitudinal displacements of monitoring point A are shown in Fig 2. The errors of the horizontal and longitudinal displacements of the monitoring point can be seen intuitively, which shows that in the foundation pit monitoring project, digital close-range photogrammetry is feasible for the measurement and optimization of the monitoring point center in combination with the error compensation methods, which guarantees the accuracy of subsequent deformation prediction.

**Fig 1:** Identification and positioning optimization results of the monitoring point center (A is the original foundation pit image; B is the optimized foundation pit image; photo taken at the Country Garden Bay International Commercial Project site in Dongguan City, Guangdong Province, China).

**Fig 2:** Changes in horizontal and longitudinal displacements at monitoring point A (A is the horizontal displacement; B is the longitudinal displacement).

### 3.2 Prediction results of deformation and displacement of foundation pits

The prediction results of the deformation displacement of the foundation pit are shown in Fig 3. In the horizontal displacement prediction, the error of the horizontal displacement predicted by the simple horizontal displacement feature is 0.35 mm at the maximum, and the error of the horizontal displacement predicted by the combination of the horizontal and longitudinal displacement features is between 0.13–0.29 mm. The error of predicting the longitudinal displacement by the simple longitudinal displacement feature is 0.24 mm at the maximum, and the error of predicting the longitudinal displacement by combining the horizontal and longitudinal displacement features is between 0–0.14 mm. Therefore, compared with the simple horizontal displacement feature and the simple longitudinal displacement feature, the prediction result, obtained by simultaneously using horizontal displacement and longitudinal displacement as input features, has smaller errors; also, the actual output is closer to the expected output.

RETRACTED

**Fig 3:** Deformation prediction results of foundation pit deformation (A is the prediction error of horizontal displacement; B is the prediction error of longitudinal displacement).

During the excavation of the foundation pit, excavation unloading in the pit will cause the structure to shift under the pressure difference between the internal and external parts, causing deformation of the external soil structure surrounding the foundation pit, and finally making the foundation pit to settle or move [20]. Therefore, it is not comprehensive to consider only horizontal displacement features or vertical displacement features. The results of this study show that the horizontal and vertical displacements are used as input features to obtain better prediction results, indicating that both the horizontal and vertical displacement features are valid input features of the neural network.

### 3.3 Prediction results of a multi-order spatiotemporal foundation pit deformation

The results of the foundation pit deformation prediction are shown in Fig 4 and Table 1. The prediction result of the feature approaches the expected output value. Among the three input features, the prediction result of the combination of time domain and space domain has the smallest RMSE, the largest IA value, and the shortest training time. Therefore, both time domain features and space domain features are valid input features of neural networks.

**Fig 4:** Prediction results of the foundation pit deformation prediction models (A is the prediction result under different input features of the BPNN model; B is the prediction result under different input features of the BPNN model optimized by the GA).

**Table 1:** Prediction results of foundation pit deformation by prediction models.

Foundation pit deformation prediction models	Input features	RMSE	IA	Training time (s)
BPNN model	Time domain	0.1043	0.8787	30.65
	Space domain	0.1445	0.8503	25.42
	Combination of time and space domains	0.0458	0.9149	23.01
BPNN model optimized by GA	Time domain	0.0669	0.8998	6.87
	Space domain	0.7950	0.9020	7.79
	Combination of time and space domains	0.0163	0.9800	7.08

In the GA-optimized BPNN model, compared with the prediction result with time domain and space domain as input features, the prediction result with time-space domain as input features is closer to the expected output. In addition, the time domain and space domain prediction results have the lowest RMSE values and the largest IA values.

RETRACTED

Taking the combination of time and space domains as input features, compared with the BPNN model, the GA-optimized BPNN model has a lower Root Mean Squared Error (RMSE) value (0.0163), a larger Index of Agreement (IA) value (0.9800), and a shorter training time (7.08 s). It shows that the GA-optimized BPNN model improves the prediction accuracy and convergence speed.

Generally, the deformation and displacement prediction of foundation pits only consider the influence of time series factors; however, for the displacement of monitoring points, both time and space characteristics are importantly related, and both have Markovian characteristics [21]. In this study, the time domain and space domain features are combined to obtain a more accurate prediction result, indicating that both time domain features and space domain features are valid input features of the neural network. Therefore, the input features need to consider not only the impact of the current monitoring point time series but also the impact of spatially adjacent monitoring points. Compared with the BPNN model, the GA-optimized BPNN model has better prediction performance. This is because the BPNN model is liable to fall into the local optimal solution when selecting the initial weights and thresholds. After it is optimized by GA, it effectively prevents convergence to the local optimal solution, overcomes the shortcomings of the BPNN model, and obtains better predictions.

### 3.4 Comparison results with other typical prediction methods

The comparison results between the GA-improved BPNN model and other typical prediction methods are shown in Fig 5. The predicted results of the SVR model and RF model have larger errors compared to the expected output values, while the GA-improved BPNN model has smaller errors and is consistent with the expected output values. The error between the prediction results of the three models and the expected output value is particularly obvious in Fig 5B. The prediction error of the SVR model is about 0.3 mm at the maximum, the prediction error of the RF model is mostly more than 0.1 mm, and the GA-optimized BPNN model has a prediction error that fluctuates between -0.06–0.09 mm. Therefore, the prediction error of the BPNN model improved by the GA is smaller than that of the SVR model and the RF model. Therefore, compared with the SVR model and the RF model, the GA-optimized BPNN has higher prediction accuracy. The comparison of prediction accuracy performance is shown in Table 2. Compared with the SVR model and RF model, the genetic algorithm-optimized BP neural network model has a lower Root Mean Squared Error (RMSE) value (0.0211), a larger Index of Agreement (IA) value (0.9706), and a shorter training time (7.61 s), indicating that the GA-improved BPNN model has more accurate prediction results.

RETRACTED

**Fig 5:** Comparison of GA-improved BPNN model and other typical prediction methods (A: Comparison of horizontal displacement; B: Comparison of horizontal displacement error).

**Table 2:** Prediction results of foundation pit deformation prediction model.

Foundation pit deformation prediction models	RMSE	IA	Training time (s)
SVR model	0.2556	0.8369	10.84
RF Model	0.3478	0.7841	10.35
GA-optimized BPNN	0.0211	0.9706	7.61

The essence of the SVM algorithm is to solve the quadratic programming problem. Therefore, problems such as slow algorithm training speed will occur when processing large sample data [22]. There are fewer parameters to be adjusted in the RF model, and its final result is the average of the results of each decision tree [23]. Therefore, the prediction errors of the SVR model and the RF model are large, and the training time is long. The GA-optimized BPNN model optimizes the performance of the combination of network weights and thresholds; therefore, the network output error is small, and its prediction result is closer to the actual value of the foundation pit deformation. The train function is used to train the BPNN, which determines the learning algorithm through adaptive adjustment, thereby improving the convergence speed of the BPNN. Therefore, the GA-optimized BPNN model has better prediction performance.

## 4. Conclusion

This study uses digital close-range photogrammetry technology to obtain monitoring data, error compensation methods to optimize the center of the monitoring point, and GA to optimize and improve the shortcomings of the BPNN algorithm. The optimized BPNN algorithm is obtained and applied in predicting the foundation pit deformation. In combination with the horizontal displacement and the longitudinal displacement, the deformation and displacement of the foundation pit is forecasted. Taking the time domain and the space domain as input features, the accuracy and efficiency of the foundation pit deformation monitoring prediction model can be improved. Therefore, the foundation pit deformation prediction model based on BPNN and GA proposed in this study has strong prediction ability, which can be applied to similar projects. This study has provided theoretical significance and application value for foundation pit deformation monitoring in geotechnical engineering, which is critical. However, the deficiencies are found in the researching process. For example, this study only compares the GA-optimized BPNN model with a simple BPNN model. Models of other algorithms combined with BPNN are not considered. Therefore, in the subsequent study, the combination of other algorithms and BPNN will be comprehensively considered, as well as the popular algorithms in artificial intelligence algorithms. Therefore, the results will be more valuable.

RETRACTED

## Supporting information

S1 Data (RAR)
